The article "Evaluation of a single‐scan protocol for radiochromic film dosimetry" was published in 2015. Journal: J Appl Clin Med Phys.

# Evaluation of a single‐scan protocol for radiochromic film dosimetry

**DOI:** 10.1120/jacmp.v16i2.5226

**Published:** 2015-03-08

**Authors:** Yoshinobu Shimohigashi, Fujio Araki, Masato Maruyama, Yuji Nakaguchi, Satoshi Kuwahara, Nozomu Nagasue, Yudai Kai

**Affiliations:** ^1^ Department of Radiological Technology Kumamoto University Hospital Kumamoto Japan; ^2^ Graduate School of Health Sciences, Kumamoto University Kumamoto Japan

**Keywords:** Gafchromic EBT3, radiochromic film dosimetry, quality assurance, intensity‐modulated radiation therapy (IMRT), multichannel

## Abstract

The purpose of this study was to evaluate a single‐scan protocol using Gafchromic EBT3 film (EBT3) by comparing it with the commonly used 24‐hr measurement protocol for radiochromic film dosimetry. Radiochromic film is generally scanned 24 hr after film exposure (24‐hr protocol). The single‐scan protocol enables measurement results within a short time using only the verification film, one calibration film, and unirradiated film. The single‐scan protocol was scanned 30 min after film irradiation. The EBT3 calibration curves were obtained with the multichannel film dosimetry method. The dose verifications for each protocol were performed with the step pattern, pyramid pattern, and clinical treatment plans for intensity‐modulated radiation therapy (IMRT). The absolute dose distributions for each protocol were compared with those calculated by the treatment planning system (TPS) using gamma evaluation at 3% and 3 mm. The dose distribution for the single‐scan protocol was within 2% of the 24‐hr protocol dose distribution. For the step pattern, the absolute dose discrepancies between the TPS for the single‐scan and 24‐hr protocols were 2.0±1.8 cGy and 1.4±1.2 cGy at the dose plateau, respectively. The pass rates were 96.0% for the single‐scan protocol and 95.9% for the 24‐hr protocol. Similarly, the dose discrepancies for the pyramid pattern were 3.6±3.5 cGy and 2.9±3.3 cGy, respectively, while the pass rates for the pyramid pattern were 95.3% and 96.4%, respectively. The average pass rates for the four IMRT plans were 96.7%±1.8% for the single‐scan protocol and 97.3%±1.4% for the 24‐hr protocol. Thus, the single‐scan protocol measurement is useful for dose verification of IMRT, based on its accuracy and efficiency.

PACS number: 87.55.Qr

## I. INTRODUCTION

Because radiochromic films exhibit useful characteristics, such as high spatial resolution, near tissue equivalence,^(1)^ and weak energy dependence,^(2)^ they are used for dose verification of intensity‐modulated radiation therapy (IMRT),^3^, ^4^ and volumetric‐modulated arc therapy (VMAT).^(5)^ Gafchromic EBT3 film (Ashland ISP Advanced Materials, NJ, USA),^(6)^ which is a commercially available radiochromic film that was recently released, comprises an active layer (28 μm thickness) sandwiched between two layers of polyester substrate (120μμm thickness) with a symmetrical structure. The surface of the polyester substrate is treated with microscopic silica particles to reduce Newton's Rings artifacts. The EBT3 film has improved structure and performance compared to the previously developed EBT and EBT2 films.^7^, ^8^, ^9^

Radiochromic film dosimetry with a color flatbed scanner provides a color channel selection option. Normally, radiochromic film dosimetry is performed with a single‐channel method using the red color channel, which has superior sensitivity to low‐dose regions.^(10)^ However, the single‐channel method may suffer from artifacts such as thickness variations of the film active layer, nonuniform scanner response, and fingerprints.^11^, ^12^ Recently, Micke et al.^(13)^ proposed a multichannel method that uses all three color channels: red, green, and blue. This method allows the separation of the dose‐dependent and dose‐independent parts of the scanned signal, and the multichannel method shows a significant improvement in spatial homogeneity. Hayashi et al.^(14)^ and Van Hoof et al.^(15)^ reported on the usefulness of the multichannel method compared to the single‐channel method. Moreover, Pevez Azorin et al.^(16)^ developed an improved multichannel method by considering the information on unirradiated film.

The postirradiation darkening of the radiochromic film is continuous with time,^7^, ^10^ and there is a 6% change in EBT2 film optical density between postirradiation times of 45 min and 24 hr.^(7)^ Therefore, the calibration film and the measurement film are scanned at the same postirradiation time in order to verify the absolute dose. A commonly used film measurement protocol is scanning of the film 24 hr after the film darkening has stabilized (24‐hr protocol).^8^, ^17^ However, an efficient film measurement protocol is required, because of the increase in the commissioning work for the treatment planning system (TPS), and because of the demand for patient‐specific quality assurance (QA) for IMRT and VMAT. Recently, Lewis et al.^(18)^ have established a new measurement protocol that combines calibration and measurement in a single scan, the so‐called single‐scan protocol. The single‐scan protocol enables measurement results within a short time using only the verification film, one calibration film, and unirradiated film. The calibration film is irradiated with a known dose at a minimum of two points (one point being unirradiated) after the irradiation of the verification film, and is used to rescale the film calibration curve.

There are few reports on clinical assessments with the single‐scan protocol using EBT3 film. Therefore, it is necessary to compare this protocol with the commonly used 24‐hr protocol, and assess its efficiency and measurement accuracy. This study aims to evaluate the single‐scan protocol using EBT3 film by comparing it with the 24‐hr protocol for dose verification of a step pattern, pyramid pattern, and clinical IMRT plans. The measurement protocol for this study was performed following the dosimetry protocol of Micke et al.^(13)^ and the approach of Lewis et al.,^(18)^ which are both included in the application software.

## II. MATERIALS AND METHODS

The film used in this study was Gafchromic EBT3 film (Lot #: 07221302) with sheet dimensions of $20.3\times 25.4\;{\text{cm}}^{2}$. The film was handled in conformance with the American Association of Physicists in Medicine (AAPM) TG‐55 report.^(1)^ All films were irradiated with 6 MV or 15 MV photons on a Clinac iX linac (Varian Medical Systems, Palo Alto, CA) and scanned after irradiation with a flatbed scanner (ES‐10000G, Seiko Epson Corp., Nagano, Japan) in transmission mode with 16 bit per color channel depth, 72 dpi resolution, and portrait orientation. The measurement and analysis of the scanned images were performed with the FilmQApro 2013 software (Ashland ISP Advanced Materials). This application is capable of analyzing both the multichannel method and the single‐scan protocol, as described in the Materials and Methods subsections A to C below. The test patterns and clinical IMRT plans were created using Eclipse version 8.9 TPS (Varian Medical Systems) with the anisotropic analytical algorithm (AAA). The TPS calculation grid size was 2.5 mm, and the benchmark of this study is the dose distribution calculated by the TPS. In order to validate the TPS, the dose profiles calculated using test patterns were checked by comparison with those given by Monte Carlo (MC) simulations. Note that the test pattern dose profiles were calculated using the EGSnrc/BEAMnrc^19^, ^20^ and DOSXYZnrc^(21)^ user codes. Incident photon particles were derived from treatment head simulations with a 6 MV photon beam, and the energy threshold and cutoff were AE=ECUT=0.7 MeV MeV and AP=PCUT=0.01 MeV, respectively. All doses were calculated with an uncertainty of within ±0.5%.

### A. EBT3 film calibration curve

The EBT3 films were cut to a size of $6\times 6\;{\text{cm}}^{2}$, and the orientation of each film was marked. The film pieces were placed at a depth of 10 cm in a $30\times 30\times 20\;{\text{cm}}^{3}$ Solid Water phantom (Gammex RMI, Middelton, WI) and irradiated with 6 MV photons with a field size of $10\times 10\;{\text{cm}}^{2}$ and source–axis distance (SAD) of 100 cm. To create a characteristic curve, films were irradiated at the dose ranges of 0, 0.25, 0.5, 0.75, 1, 1.25, 1.5, 1.75, 2, 2.5, 3, 3.5, 4, 6, 8, and 10 Gy. The absolute dose was measured at the same depth as the film using a 0.6 cm^3^ Farmer ionization chamber (TN30013, PTW Freiburg, Germany). The irradiated EBT3 films were scanned 24 hr postirradiation. The optical density (OD) of the scanned film images was measured by setting a $5\times 5\;{\text{cm}}^{2}$ region of interest (ROI) at the center of each image. The calibration curve of the EBT3 film using FilmQApro was fitted to the following rational function:(13)

(1) $$d_{x,D}(D)=-{\text{log}}_{10}((a_{x}+b_{x}D)/(c_{x}+D))$$

where *x* is the color channel (red, green, or blue); $d_{x,D}(D)$ is the calibration function of the x channel; *D* is the dose; and *a, b*, and *c* are parameters of the function.

### B. Film dosimetry using the multichannel method

The multichannel method uses the following formula to model the film calibration curve, which separates the dose‐dependent part of the scanned OD from any disturbance, $\Delta d_{x}$, such as film nonuniformity, nonuniform scanner response, fingerprints, and other error factors:^(13)^

(2) $$d_{x,\text{scan}}(D)=d_{x,D}(D)\Delta d_{x}$$

where $d_{x,D}(D)$ is the calibration function of the x channel and $d_{x,scan}(D)$ is the scanned single pixel OD for the same x channel.

Here, $\Delta d_{x}$ is calculated using the method of least squares to minimize the difference in the dose results from the three color channels (red, green, and blue):^(13)^

(3) $$\text{min}\Delta d_{\left(R,G,B\right)}={\left(\Delta d_{R}-\Delta d_{B}\right)}^{2}+{\left(\Delta d_{B}-\Delta d_{G}\right)}^{2}+{\left(\Delta d_{G}-\Delta d_{R}\right)}^{2}$$

The above calculations are performed automatically by selecting the multichannel method in FilmQApro.

### C. Single‐scan measurement protocol

The single‐scan protocol in this study was performed using the verification film, one calibration film, and unirradiated film. The EBT3 film was cut to $20.3\times 20.3\;{\text{cm}}^{2}$ square to create for the verification film, while the remaining $20.3\times 5.1\;{\text{cm}}^{2}$ strip was used as the calibration and unirradiated films. The verification film was placed at a depth of 10 cm in a $30\times 30\times 20\;{\text{cm}}^{3}$ Solid Water phantom and irradiated according to the test patterns and clinical IMRT plans. The calibration film was used to rescale the calibration curve of the film and was irradiated at two points with a known dose in an arrangement similar to that of the verification film. One point was unirradiated (0 Gy), and the other point was irradiated with 3 Gy, which is 1.5 times the verification dose range (∼2 Gy). A single calibration film is required for all verification film. The calibration film and verification film were irradiated within a narrow time window and were scanned 30 min later, so as to reduce dose errors caused by postirradiation changes in the film.^(18)^ Figure 1 shows the film‐scanning arrangement in the single‐scan protocol.

**Figure 1:** Film‐scanning arrangement in the single‐scan protocol: (a) verification film; (b) unirradiated film; (c) calibration film.

### D. Evaluation of the measurement protocol for the dose verification of step pattern, pyramid pattern, and clinical IMRT plans

The single‐scan protocol was evaluated through comparison with the commonly used 24‐hr protocol. As shown in Fig. 2, the dose patterns used for the verification were a step pattern composed of four striped steps with dose levels of 0.6, 1.1, 1.6, and 2 Gy, and a pyramid pattern with dose levels of 0.7, 1.3, and 2 Gy. The films were placed at a depth of 10 cm in a $30\times 30\times 20\;{\text{cm}}^{3}$ solid water phantom at a SAD of 100 cm and irradiated with 6 MV photons at a gantry angle of 0°. The irradiated EBT3 films were scanned after 30 min and 24 hr for the single‐scan and the 24‐hr protocols, respectively. The two‐dimensional (2D) dose distributions obtained by each protocol were compared with those of the TPS and evaluated by the gamma analysis method.^22^, ^23^ The dose profiles were acquired along the arrows in Fig. 2. An ROI encompassing the area approximately 10 mm from the film edge was defined and the number of points satisfying the condition Γ<1 was calculated using the global gamma. The TPS‐calculated dose distributions were linearly interpolated to a grid size of 1 mm for gamma evaluation. The gamma evaluation was performed with a tolerance level of 3% and 3 mm, which are the dose difference (DD) and distance‐to‐agreement (DTA) values, respectively, with a 30% threshold (TH) to exclude the low‐dose region. The tolerance level of DD was calculated relative to the maximum dose.

The dose verifications of the clinical IMRT plans were used to further evaluate the single‐scan protocol. The parameters of the clinical IMRT are listed in Table 1. We delivered four IMRT plans (head, neck, pelvis, prostate) and compared the measured dose with the calculated dose distributions from the TPS. Depending on the IMRT plans, the maximum doses delivered to the verification film ranged from approximately 1.8 Gy to approximately 2 Gy. The clinical IMRT plans were performed at a film position with a phantom similar to the step and pyramid patterns. Scanning and analysis of the irradiated EBT3 films were the same as those for the step and pyramid pattern; the overall uncertainty of the EBT3 film measurement was estimated using the method proposed by van Battum et al.^(24)^ The overall uncertainty was estimated to be 2%.

**Figure 2:** EBT3 film response with dose pattern used for the verification: (a) step pattern composed of four striped steps with dose levels of 0.6, 1.1, 1.6, and 2 Gy; and (b) pyramid pattern with dose levels of 0.7, 1.3, and 2 Gy. The dose profiles were acquired along the *white arrows* at a depth of 10 cm in a Solid Water phantom.

**Table 1:** Parameters of clinical IMRT plans calculated with Eclipse TPS

*Plan No.*	*Energy*	*Treatment Site*	*Gantry Angle (θ)*	*Dose (Gy)/Fraction*
1	6 MV	Head	35°, 95°, 150°, 225°, 285°, 290°	2.0
2	6 MV	Neck	60°, 105°, 150°, 180°, 210°, 255°, 300°	1.8
3	6 MV	Pelvis	25°, 75°, 125°, 180°, 235°, 285°, 335°	1.8
4	15 MV	Prostate	35°, 105°, 180°, 225°, 325°	2.0

## III. RESULTS

### A. Dose verification of the step and pyramid patterns

Figure 3 shows the comparison of the dose profiles with the step and pyramid pattern for the single‐scan protocol, 24‐hr protocol, TPS, and MC simulation. The TPS‐calculated dose profile agreed within 2% with the MC‐calculated results, while the dose profiles for the single‐scan also agreed within 2% with those of the 24‐hr protocol. For the step pattern, the absolute dose discrepancies from the TPS for the single‐scan and 24‐hr protocols were 2.0±1.8 cGy and 1.4±1.2 cGy at the low‐dose gradient, respectively. Similarly, the dose discrepancies for the pyramid pattern were 3.6±3.5 cGy and 2.9±3.3 cGy, respectively. Figure 4 shows the comparison of the 2D dose distributions with the step and pyramid pattern for the single‐scan protocol, 24‐hr protocol, and TPS. The dose distributions for each protocol agreed well with those of the TPS. Table 2 summarizes the results of gamma analysis for a DD of 3% and DTA of 3 mm. The gamma pass rates for the single‐scan protocol were 96.0% and 95.3% for the step and pyramid pattern, respectively. The gamma pass rates for the 24‐hr protocol for the step and pyramid pattern were 95.9% and 96.4%, respectively.

**Figure 3:** Comparison of the dose profiles with (a) step and (b) pyramid pattern for the single‐scan protocol, 24‐hr protocol, Eclipse‐TPS, and MC simulation. The dose profiles were acquired at a depth of 10 cm in a Solid Water phantom.

**Figure 4:** Comparison of 2D dose distributions with the step and pyramid pattern for the single‐scan protocol, 24‐hr protocol, and Eclipse‐TPS. The dose distributions were acquired at a depth of 10 cm in a Solid Water phantom. Dose distribution with step pattern: dose distributions calculated from (a) single‐scan protocol (thin lines), (b) 24‐hr protocol (thin lines) and Eclipse‐TPS (thick lines). Dose distribution with pyramid pattern: dose distributions calculated from (c) single‐scan protocol (thin lines), (d) 24‐hr protocol (thin lines) and Eclipse‐TPS (thick lines).

**Table 2:** Comparison of gamma analysis with the dose difference of 3% and distance‐to‐agreement of 3 mm for varying the dose patterns. The gamma analysis was conducted using the global gamma with a 30% threshold. The absolute dose difference between the measured and Eclipse TPS‐calculated dose is listed in the brackets

*Dose Pattern*	*Gamma Pass Rate (3%, 3 mm) (Absolute Dose Difference: cGy)* ^a^	
	*Single‐scan Protocol*	*24‐hr Protocol*
Step	96.0% (2.0±1.8 cGy)	95.9% (1.4±1.2 cGy)
Pyramid	95.3% 96.4% (3.6±3.5 cGy)	(2.9±3.3 cGy)

^a^ Absolute dose difference is presented as the average ±1 SD.

### B. Dose verification of clinical IMRT plan

Figure 5 shows the comparison of the 2D dose distributions with the neck and prostate IMRT plans for the single‐scan protocol, 24‐hr protocol, and TPS. The dose distributions for each protocol agreed well with those of the TPS. Figure 6 shows the comparison of the dose profiles with the neck and prostate IMRT plans for the single‐scan protocol, 24‐hr protocol, and TPS. For the neck IMRT plan, the absolute dose discrepancies from the TPS for the single‐scan and the 24‐hr protocol were 2.5±2.7 cGy and 2.7±2.5 cGy at the low‐dose gradient, respectively. Similarly, the dose discrepancies for the prostate IMRT plan were 3.8±3.8 cGy and 3.6±2.3 cGy, respectively. The results of the dose profile for other IMRT plans were also similar to those for the neck and prostate IMRT plans. Table 3 summarizes the results of the four IMRT plans for gamma analysis with a DD of 3% and DTA of 3 mm. The average pass rates were 96.7%±1.8% for the single‐scan protocol and 97.3%±1.4% for the 24‐hr protocol. The total time interval to deliver the IMRT plan was dependent on the treatment sites, while the beam delivery times were within 5 min for the head and prostate plans, and within 10 min for the neck and pelvis plans. The calibration film for the single‐scan protocol was irradiated within 5 min. The total time interval for the single‐scan protocol was within 20 min, including the phantom setup. However, the total time interval required to deliver the IMRT plan may not be sufficiently short with respect to the 30‐min postexposure reading time gap.

**Figure 5:** Comparisons of 2D dose distributions with neck and prostate IMRT plan for the single‐scan protocol and the 24‐hr protocol and Eclipse‐TPS. The dose distributions were acquired at the depth of 10 cm in a Solid Water phantom. Dose distribution with neck IMRT plan: dose distributions calculated from (a) single‐scan protocol (thin lines), (b) 24‐hr protocol (thin lines) and Eclipse‐TPS (thick lines). Dose distribution with prostate IMRT plan: dose distributions calculated from (c) single‐scan protocol (thin lines), (d) 24‐hr protocol (thin lines) and Eclipse‐TPS (thick lines).

**Figure 6:** Comparisons of the dose profiles with (a) neck and (b) prostate IMRT plan for the single‐scan protocol, the 24‐hr protocol, and Eclipse‐TPS. The dose profiles were acquired along the *arrows* in Fig. 5 at a depth of 10 cm in a Solid Water phantom.

**Table 3:** Comparison of gamma analysis with the dose difference of 3% and distance‐to‐agreement of 3 mm for the four clinical IMRT plans. The gamma analysis was conducted using the global gamma with a 30% threshold

*Plan No.*	*Gamma Pass Rate (3%, 3 mm)*	
	*Single‐scan Protocol*	*24‐hr Protocol*
1	99.0%	98.5%
2	95.5%	97.4%
3	95.3%	95.3%
4	97.8%	97.8%

## IV. DISCUSSION

Radiochromic film dosimetry was conducted with the multichannel method using EBT3 film. The EBT3 film calibration curves showed results similar to those of other reports.^4^, ^7^, ^8^, ^10^ The red channel had a high sensitivity in the clinical dose range,^4^, ^10^ the green channel showed potential for use in higher dose ranges,^(7)^ while the blue channel was the most insensitive due to the effect of the yellow marker dye.^(8)^ The dose values for the multichannel method were calculated using all three color channels. The dose profiles for the 24‐hr protocol using the multichannel method agreed within 3% with those of the TPS, and the average dose discrepancies were less than 5 cGy at the low‐dose gradient. Furthermore, the gamma pass rates with a DD of 3% and DTA of 3 mm were over 95% for all plans. Van Hoof et al.^(15)^ assessed the multichannel method using EBT2 film and reported that the dose discrepancies from the TPS were small, in the order of 0 to 5 cGy for a single square beam. Hayashi et al.^(14)^ also performed a similar assessment and reported that the average gamma pass rates in the IMRT and VMAT dose verification were 97.2%±0.8%. The results from the multichannel method in this study showed a similar trend. Recently, Azorin et al.^(16)^ proposed an improved method for multichannel dosimetry, which considers information from unirradiated film. This method improved the gamma analysis results for the IMRT dose verification compared with the other multichannel methods. The pass rates results with a DD of 3% and DTA of 3 mm for 30 IMRT verifications were 97.8%±2.0% and 96.0%±2.6% for the improved method and Micke et al.^(13)^ methods, respectively.

This study evaluated the measurement accuracy of the single‐scan protocol by comparing IMRT dose verification with the 24‐hr protocol. Our study performed dose verification for the test patterns and four clinical IMRT plans. For the single‐scan protocol, a single calibration film was irradiated for all verification film. The dose profiles and gamma pass rates for the single‐scan protocol were consistent with those of the 24‐hr protocol, owing to the adjustment of the calibration curve using the calibration film in the single‐scan protocol. Note that the only difference between the two measurement protocols is the rescaling factor. Lewis et al.^(18)^ established the single‐scan protocol and assessed its efficacy with the IMRT and VMAT plans for 6 MV photons at limited treatment sites. They reported that the gamma pass rates with a DD of 2% and DTA of 2 mm were over 97%. Our study applied the single‐scan protocol to IMRT plans for various treatment sites and two‐photon energy, which showed a trend similar to that reported by Lewis et al.^(18)^ Moreover, it is known that the radiochromic film response varies slightly with respect to photon energy, temperature, and humidity.^1^, ^2^ However, the results of our study did not sufficiently support the conclusion that the differences in the film response were caused by the photon energy and measurement environment.

Recently, several reports pertaining to efficient measurement methods for radiochromic film dosimetry were published. Devic et al.^(10)^ described a procedure by which one can establish an acceptable time window around the chosen postirradiation scanning time protocol that would provide an acceptable dose error. They showed that a 1% dose error could be achieved if the scanning time window were less than ±5 min for the 30‐min protocol and ±2 hr for the 24‐hr postirradiation scanning time protocols. However, as a matter of clinical practice, it is difficult to achieve a scanning time window within ±5 min for the 30‐min protocol. Furthermore, Devic et al.^(25)^ demonstrated the use of a functional argument to linearize the inherently nonlinear response of a radiochromic film‐based reference dosimetry system, and showed that relative dosimetry can be conveniently performed using a radiochromic film dosimetry system without establishing a calibration curve. The radiochromic film response to the postirradiation time is not important for the measurement of relative dose, but it is important for the absolute dose. The dose verifications for the single‐scan protocol were scanned 30 min after film irradiation, and the measurement accuracy was within 3% of the absolute dose. Chang et al.^(26)^ proposed a film calibration method that includes the effect of the postirradiation time, ranging from 1 h to two months. The accuracy of the film doses for delivered doses above 60 cGy were mainly within 2% and the total uncertainties were generally less than 5%. The efficient measurement method must be selected whether the verification is performed for a relative or absolute dose.

The dose verifications for the single‐scan protocol in this study allow for measurement 30 min postirradiation using one calibration film and unirradiated film. However, the single‐scan protocol can be applied at any time, although our results have not been examined in sufficient detail in that respect. Moreover, this study did not evaluate film lot differences, multiplanar irradiation, or dose verification of VMAT plans. However, from the results of dose verification with IMRT plans in this study, the single‐scan protocol is clinically useful because of its measurement accuracy and efficiency.

## V. CONCLUSIONS

This study evaluated the single‐scan protocol using EBT3 film by comparing it with the commonly used 24‐hr protocol for the dose verification of the step pattern, pyramid pattern, and clinical IMRT plans. The dose verification for the single‐scan protocol showed measurement accuracy similar to that of the 24‐hr protocol, demonstrating that it is clinically useful for efficient IMRT dose verification.

## ACKNOWLEDGMENTS

The authors would like to thank the VERITAS Corporation in Japan for their helpful comments.
